RETRACTED

# Overexpression of NTRK1 Promotes Differentiation of Neural Stem Cells into Cholinergic Neurons

**DOI:** 10.1155/2015/857202

**Published:** 2015-10-05

**Authors:** Limin Wang, Feng He, Zhuoyuan Zhong, Ruiyan Lv, Songhua Xiao, Zhonglin Liu

**Affiliations:** ^1^Department of Neurology, Guangdong General Hospital, Guangdong Academy of Medical Sciences, Guangdong Neuroscience Institute, Guangzhou, Guangdong 510080, China; ^2^Department of Neurology, Linyi City People's Hospital, Linyi, Shandong 276000, China; ^3^Guangdong Provincial Key Laboratory of Malignant Tumor Epigenetics and Gene Regulation, Department of Neurology, Sun Yat-sen Memorial Hospital, Sun Yat-sen University, Guangzhou, Guangdong 510120, China

## Abstract

Neurotrophic tyrosine kinase type 1 (NTRK1) plays critical roles in proliferation, differentiation, and survival of cholinergic neurons; however, it remains unknown whether enhanced expression of NTRK1 in neural stem cells (NSCs) can promote their differentiation into mature neurons. In this study, a plasmid encoding the rat NTRK1 gene was constructed and transfected into C17.2 mouse neural stem cells (NSCs). NTRK1 overexpression in C17.2 cells was confirmed by western blot. The NSCs overexpressing NTRK1 and the C17.2 NSCs transfected by an empty plasmid vector were treated with or without 100 ng/mL nerve growth factor (NGF) for 7 days. Expression of the cholinergic cell marker, choline acetyltransferase (ChAT), was detected by florescent immunocytochemistry (ICC). In the presence of NGF induction, the NSCs overexpressing NTRK1 differentiated into ChAT-immunopositive cells at 3-fold higher than the NSCs transfected by the plasmid vector (26% versus 9%, *P* < 0.05). The data suggest that elevated NTRK1 expression increases differentiation of NSCs into cholinergic neurons under stimulation of NGF. The approach also represents an efficient strategy for generation of cholinergic neurons.

## 1. Introduction

The family neurotrophic tyrosine receptor kinase (NTRK), also known as tropomyosin receptor kinases (Trk), includes receptors regulating synaptic strength and plasticity in the mammalian nervous system [1]. NTRK1 is one of the three major family members. NTRK1 is synthesized in basal forebrain cholinergic neurons (BFCN) and displayed on their axons, where NTRK1 is bound by its primary ligand, nerve growth factor (NGF) [2, 3]. Expression of NTRK1 precedes expression of choline acetyltransferase (ChAT), the enzyme that mediates the biosynthesis of acetylcholine and serves as a marker of cholinergic neurons, during the development of central nervous system (CNS) [4, 5]. NGF produced by neocortical neurons can experimentally induce basal forebrain cells to differentiate into cholinergic cells through activation of NTRK1 [6–10]. Hence, NTRK1 is considered to be involved in the early neuronal development.

RETRACTED

NTRK1 is synthesized in BFCN from development to adulthood [5] and is necessary for NGF-mediated survival of the neurons [11]. BFCNs are the predominant source of cortical cholinergic input and play a central role in spatial learning and memory [12]. Loss of these neurons parallels cognitive decline and is associated with Alzheimer's disease (AD) [13], a progressive debilitating neurodegenerative disorder that typically occurs in the elderly. Postmortem examination of the brains of patients diagnosed with early stage AD has shown that NTRK1 expression is reduced in BFCN [14], indicating that downregulation of NTRK1 contributes to the loss of the neurons and the early onset of AD. In addition, genetic variants of neurotrophin system genes including NTRK1 have been found to confer susceptibility to AD [15].

Although increasing evidence suggests NTRK1 plays critical role in proliferation, differentiation, and survival of cholinergic neurons [16–19], it remains unknown whether enhanced expression of NTRK1 in neural stem cells (NSCs) can promote their differentiation into mature neurons.

In this study, we transfected mouse NSCs (C17.2 cell line) with a plasmid encoding the NTRK1. Under induction of NGF, the NCSs overexpressing NTRK1 differentiated into cholinergic neurons at 3-fold higher efficiency than the NCSs transfected by an empty vector. To the best of our knowledge, this is the first direct evidence from cell culture to show that enhanced expression of NTRK1 promotes the differentiation of NSCs under stimulation of NGF.

## 2. Materials and Methods

### 2.1. Construction of Plasmid Encoding NTRK1

Total RNA was isolated from PC12 cell line which is derived from a pheochromocytoma of the rat adrenal medulla. NTRK1 cDNA was synthesized by reverse transcription polymerase chain reaction (RT-PCR) using oligo (dT) primer according to the manufacturer's instructions. The NTRK1 gene was amplified by PCR using primers 5′-tctgaattcatgctgcgaggccagcggca-3′ and 5′-actctcgagctagcccagaacgtccaggt-3′. The amplified NTRK1 gene was digested by EcoRI and XhoI at restriction sites introduced by the primers. The digested NTRK1 gene was then purified and cloned into plasmid vector pcDNA3.1(+) digested with the same enzymes. The resulting plasmid pcDNA-NTRK1 was confirmed by DNA sequencing.

### 2.2. Cell Culture and Transfection

The mouse C17.2 neural stem cells preserved in our laboratory were seeded in 6-well plates at a density of 1 × 10^5^ cells with Dulbecco's Modified Eagle Medium (DMEM) containing 10% fetal bovine serum (FBS) (Invitrogen, Carlsbad, CA, USA), 5% horse serum (HS) (Sigma Aldrich, St. Louis, MO, USA), and 2 mM glutamine in a humidified incubator (5% CO_2_, 95% air) at 37°C. When the cell monolayers reached a confluence of ≥70%, the cells were subjected to a transfection procedure using the Lipofectamine 2000 (GIBCO BRL company, Foster City, CA, USA) in accordance with the manufacturer's instructions. For each well of cells, 1 *μ*g of plasmid DNA and 3 *μ*L Lipofectamine 2000 were each diluted in 50 *μ*L of serum-free medium. They were combined after 10 min of incubation at room temperature (RT), and the mixture was left at RT for 45 min. The mixture was supplemented with serum-free medium until final volume of 1 mL and transferred to the cells prewashed twice with serum-free medium. After 5 h, the medium was replaced with DMEM medium containing 10% FBS and 5% HS. At two days after transfection, the cells were trypsinized and subcultured in growth media containing 200 *μ*g/mL G418. The G418-resistant clones were pooled, amplified, and maintained in the selective growth media.

RETRACTED

### 2.3. Western Blotting

Cells were lysed in RIPA buffer containing 25 mM Tris.Cl pH 7.6, 150 mM NaCl, 1% NP-40, 1% sodium deoxycholate, and 0.1% SDS. Total protein was measured using the BCA method. For each sample, 15 *μ*g of total protein was resolved by 12% sodium dodecyl sulfate polyacrylamide gel electrophoresis (SDS-PAGE) and transferred to PVDF membrane. The blots were probed with primary antibodies specific to NTRK1 (1 : 1000) or *β*-actin (1 : 1000) at 4°C overnight. The membranes were then incubated with secondary antibodies conjugated with horseradish peroxidase (HRP) for 60 min. Proteins bands were visualized using enhanced chemiluminescence (ECL) substrate and exposed to X-ray film.

### 2.4. Induction of Cellular Differentiation

The G418-resistant C17.2 cells overexpressing NTRK1 were seeded into 6-well plates and cultured in growth media with or without 100 ng/mL NGF. As control, the G418-resistant C17.2 cells without NTRK1 overexpression were also treated with the same procedure. ChAT expression was detected after 7 days of treatment.

### 2.5. Florescent Immunocytochemistry (ICC)

Cells were fixed in 4% polymethonal for 30 min, washed in phosphate buffered saline (PBS) three times, and blocked with normal goat serum (NGS) for 1 h. Subsequently, the cells were washed in PBS and incubated with rabbit anti-ChAT polyclonal antibody (Boster, Wuhan, China) at 4°C overnight. The cells were washed and incubated with goat anti-rabbit IgG FITC-conjugated secondary antibody at 32°C for 1 h. The labeled cells were observed under a fluorescence microscope (Nikon, TE2000). From 12 random fields of view, the ChAT-positive cells as well as the total cells were counted for each treatment group.

RETRACTED

### 2.6. Statistical Analysis

For each field of view, the ratio of ChAT-positive cells to total cells was calculated as the frequency of cells expressing ChAT. The average mean frequency was calculated using the frequencies obtained from 12 random fields of view. The data are presented as means ± standard deviation. The statistical analysis was performed using the Student's *t*-test as described previously [20]. *P* < 0.05 was considered statistically significant.

## 3. Results

### 3.1. NTRK1 Overexpression

The complete NTRK1 coding sequence (CDS) was amplified from PC12 rat cell line and cloned into plasmid vector pcDNA3.1(+) downstream the cytomegalovirus (CMV) promoter resulting plasmid pcDNA-NTRK1. The C17.2 neural stem cells were transfected by pcDNA-NTRK1 and empty vector pcDNA3.1(+), respectively. The G418-resistant cells were selected and expanded. The level of NTRK1 expression was measured using western blot. As shown in Figure 1, the NSCs transfected by pcDNA-NTRK1 expressed NTRK1 at much higher level than the NSCs transfected by the empty vector pcDNA3.1(+). The latter has similar level of NTRK1 as the nontransfected control C17.2 NSCs. The data confirmed that the NTRK1 gene had been successfully transfected into the NSCs.

### 3.2. Identification of Cholinergic Neurons

The NSCs proved to overexpress NTRK1 were cultured in serum-free media with or without NGF. Seven days of NGF induction resulted in efficient generation of cells expressing ChAT measured by ICC (Figure 2). As control, the G418-resistant NSCs derived from C17.2 cells transfected by the empty vector were also treated similarly. Although NGF treatment led to generation of ChAT-expressing cells, less efficient than the NSCs overexpressing NTRK1, the ChAT-negative cells included astrocytes and small round cells which may at least include nondifferentiated NSCs. From 12 random fields of view, the ChAT-positive cells and the total cells were counted. Under treatment of NGF, the percentage of ChAT-positive cells was 25.98 ± 4.71% for NSCs overexpressing NTRK1 and was 9.08 ± 3.26% for NSCs transfected by the plasmid vector (*P* < 0.01). Of note, the experiment represents three independent experiments which had consistent findings.

The ChAT positive ratio of NTRK1-transfected cells exposed to NGF was (25.98 ± 4.71)%, and that of pseudotransfected cells exposed to NGF was (9.08 ± 3.26)% (*P* < 0.01, NGF-treated NTRK1-transfected versus NGF-treated pseudotransfected exposed to NGF) (Figure 3). No fluorescent labeling was observed in either the nontransfected control cells or the NTRK1-tranfected cells that were not exposed to NGF.

RETRACTED

## 4. Discussion

Growing evidence shows that NTRK1 plays critical role in the differentiation and survival of neurons. However, it remains obscure how NTRK1 expression level in neural stem cells affects differentiation efficiency. In this study, the full length NTRK1 gene was stably transferred into neural stem cells. Overexpression of NTRK1 led to 3-fold higher differentiation efficiency (26% versus 9%) when subjected to stimulation by NGF. These findings indicate that differentiation of NSCs into a cholinergic fate is related to expression level of NTRK1.

NTRK1 (TrkA), NTRK2 (TrkB), and NTRK3 (TrkC) are the three major members of NTRK family. These three receptors together with another membrane receptor, p75NTR, play central role in the proliferation, differentiation, and survival of neurons [1]. NTRK1 is bound and activated by NGF [21, 22]. NT-3 also binds NTRK1 as a lower affinity heterologous ligand [23]. In the presence of p75NTR, NGF shows enhanced activation of NTRK1 [24–26], as p75NTR increases the rate of NGF association with NTRK1 [27]. On the other hand, NT3 becomes much less effective at activating NTRK1 due to the presence of p75NTR [28–30].* NTRK1* gene has 17 exons [31]. Different isoforms of NTRK1 also affect the neurotrophin-mediated signaling. The isoform lacking a short insert in the juxtamembrane region is activated efficiently only by NGF. Presence of this insert increases activation of NTRK1 by NT3 without affecting its activation by NGF [32]. Although the differentiation of NSCs is regulated by a complicated network* in vivo*, use of* in vitro* cultured cells allows us to determine the effect of NGF on the differentiation of NSCs without interfering by other neurotrophins, consistent with previous finding that the NSCs (C17.2 cells) synthesize NTRK1 [33], but at a much lower level compared to the cells stably transfected by plasmid encoding* NTRK1* gene. This is expected as the CMV promoter which drives the* NTRK1* gene in the plasmid has been proven highly active in neurons [34].

C17.2 is an immortalized mouse neural progenitor cell line which was established by retroviral-mediated transduction of the v-*myc* oncogene into mitotic progenitor cells of neonatal mouse cerebellum [35]. C17.2 cells are maintained as monolayer in cell culture dishes in DMEM supplemented with fetal calf serum and horse serum. Under induction of serum-free media containing neurotrophins, the C17.2 cells differentiate into neurons and astrocytes with distinct morphology. ChAT is the enzyme responsible for synthesis of acetylcholine from acetyl-coenzyme A and choline and is found in high concentration in cholinergic neurons, both in the central nervous system (CNS) and in peripheral nervous system (PNS). Our data showed that the parental C17.2 cells could be induced to differentiate into cholinergic neurons, but less efficient than the NSCs overexpressing NTKR1. This is most likely because more molecules of NTRK1 displayed on the membrane facilitate the NGF-mediated signal transduction.

RETRACTED

NTRK1 consists of an extracellular ligand-binding domain, a single transmembrane domain, and an intracellular tyrosine kinase domain. After being bound by nerve growth factor (NGF), NTRK1 is activated and initiates a signaling cascade of molecules including Ras/Raf/MAP kinase, PI3K/Akt, and PLC-*γ* [36–38]. However, it remains poorly understood how these NTRK1-activated pathways regulate the differentiation and survival of the neurons. It has been found that the cholinergic gene locus contains a region located within 2 kb immediately 5′ border of the R-exon, which confers responsiveness to NGF in reporter gene assays [39]. The region contains two activator protein 1 (AP-1) sites as well as a putative cAMP response element (CRE) [40]. However, the precise mechanism between NTRK1 activation and ChAT expression has not yet been appreciated. In this study we focused on cholinergic neurons generated under induction of NGF. But it is interesting to examine whether other types of neurons were generated during the process. Furthermore, the cholinergic neurons may also synthesize other transmitters as reported previously [41].

In conclusion, the present study demonstrated that overexpression of NTRK1 facilitates more efficient differentiation of NSCs into cholinergic neuron in response to NGF treatment. It also represents an efficient strategy to generate cholinergic neurons.

## Figures and Tables

**Figure 1:** Western blot analysis of NTRK1 expression in NSCs. NTRK1 expression was measured in the nontransfected C17.2 cells, and G418-resistant C17.2 cells derived from transfections using pcDNA-NTRK1 or the empty vector pcDNA3.1(+). *β*-actin was measured to serve as an internal loading control.

**Figure 2:** ICC photomicrographs (400x) of G418-resistant NSCs with or without NGF treatment. In the absence of NGF exposure, pcDNA3.1(+)-transfected cells (a) and pcDNA-NTRK1-transfected cells (b) showed no ChAT expression. Following NGF exposure for 7 d, both pcDNA3.1(+)-transfected cells (c) and pcDNA-NTRK1-transfected cells (d) were immunopositive for ChAT (FITC labeled).

**Figure 3:** Ratio of ChAT positive cells differentiated in the NTRK1 transfected group (D) was higher than that in the pseudotransfected group (C) (*n* = 12).
